# Effect of Comprehensive Care Based on Appropriate Chinese Medicine Techniques on Urinary Retention and Bladder Function Recovery after Total Hysterectomy in Patients with Cervical Cancer

**DOI:** 10.1155/2022/7495418

**Published:** 2022-06-30

**Authors:** Qing Lu, LiangHong Wu, LiYing Qi, Ping Tie, Zhihong Guan

**Affiliations:** ^1^Jiangsu Cancer Hospital, China; ^2^Jiangsu Institute of Cancer Disease Prevention and Control, China; ^3^Affiliated Cancer Hospital of Nanjing Medical University, China

## Abstract

**Objective:**

To investigate the effect of comprehensive care based on appropriate Chinese medicine techniques on urinary retention and bladder function recovery after total hysterectomy in patients with cervical cancer.

**Methods:**

A total of 148 cases admitted after radical hysterectomy for cervical cancer from January 2019 to early September 2019 were used as the observation sample and were divided into control and experimental groups based on a randomized double-blind method. There were 74 cases each. The control group was given comprehensive care, and the experimental group was given comprehensive care based on appropriate Chinese medicine techniques. The intervention period was 2 weeks after surgery. The recovery rate of bladder function and the occurrence of urinary retention were compared between the two groups, and the duration of postoperative retention of urinary catheter, the amount of residual urine, and the feeling of urination were counted.

**Results:**

The experimental group had better urinary catheter retention time, time to first spontaneous voiding, time to get out of bed, and time to anal discharge than the control group; the experimental group had a higher rate of good bladder function recovery than the control group and better bladder recovery time, residual urine volume, and incidence of urinary retention than the control group; the patients in the experimental group had better UDI-6 scores.

**Conclusion:**

The implementation of comprehensive care based on appropriate Chinese medicine techniques can relieve patients' difficulty in urination and improve their quality of life.

## 1. Introduction

Cervical cancer is one of the most common malignancies in gynaecology, with approximately 500,000 new cases of cervical cancer each year worldwide [1, 2]. At present, surgery is the first choice of treatment for early-stage cervical cancer [3, 4]. Radical hysterectomy+pelvic lymph node dissection is one of the conventional treatments for gynaecological malignancies [5, 6]. However, the surgery is extensive and invasive, with many postoperative complications and bladder dysfunction. Urinary retention is one of the common postoperative complications. Urinary retention is defined as the inability to pass urine for more than 15 d after surgery or the ability to pass urine on one's own but with residual urine ≥ 100 ml [7–9]. Urinary retention can have many adverse effects on patients, including quality of life, speed of recovery, and other illnesses, so it is not only important to manage it effectively, but prevention is the best medical intervention to target [10]. Long-term indwelling urinary catheters can cause urinary tract infections, which can cause pain and affect the patient's daily life, as well as affecting the patient's image and causing a certain sense of inferiority [11, 12]. These will have a serious impact on the quality of life of the patient. It is therefore particularly important to explore the impact of reducing the occurrence of urinary retention to facilitate the recovery of bladder function in patients after radical hysterectomy.

Chinese medicine classifies urinary retention as “retention of urine” and “gonorrhea” and cites pericystal vascular disease, neurological dysregulation, and toxic blockage of the bladder as important factors in triggering urinary retention [13–15]. Chinese medicine techniques such as acupuncture, acupressure, foot and umbilical therapy, and medicinal baths can effectively improve the blood circulation of the bladder vessels and provide anti-inflammatory and pain relief, laxative and diuretic effects, and relieve retention, which are of great value in clinical care [16, 17]. Snap-on needles are short for snap-on intradermal needles, which have a looped end and are perpendicular to the body of the needle, also known as stud-type intradermal needles [18]. Auricular acupressure is based on the biological holographic theory, which states that auricular acupuncture points are located in specific areas on the eardrum, which are the reaction points of the internal organs, body, and limbs of the human body on the eardrum, whereas the application of traditional Chinese medicine characteristic therapy of pressing needle+auricular point sticking and pressing is still less after radical hysterectomy. From January 2019 to early September 2019, a total of 148 patients with cervical cancer after radical hysterectomy+pelvic lymph node dissection were treated in our hospital. Through comparative observation and analysis, we explored the clinical effect of comprehensive nursing based on the appropriate technology of traditional Chinese medicine on the recovery of bladder function and the reduction of urinary retention after cervical cancer surgery. The report is as follows.

## 2. General Information

Prospectively, 148 patients admitted to our hospital from January 2019 to early September 2019 who underwent radical hysterectomy+pelvic lymph node dissection for cervical cancer were selected as the study population. The patients were divided into 74 cases each in the experimental group and control group according to the random number table method. The control group criteria are as follows: aged 35-66 years, mean (47.25 ± 5.36 years), clinical stage (25 cases of stage I and 49 cases of stage II), and pathological classification (50 cases of squamous carcinoma of the cervix and 24 cases of adenocarcinoma). The experimental group criteria are as follows: aged 34-65 years, mean (46.25 ± 5.14 years), clinical stage (28 cases of stage I and 46 cases of stage II), and pathological classification (50 cases of squamous carcinoma and 24 cases of adenocarcinoma of the cervix. The patients were treated with TCM appropriate techniques on the basis of conventional care after surgery. There were no statistically significant differences between the two groups in terms of age, clinical stage, pathological classification, and other general information (*p* > 0.05). Inclusion criteria are as follows: cervical cancer confirmed by preoperative tissue biopsy and postoperative pathology; expected postoperativesurvival > 12 months; and clinical stage Ia-IIb. The study was approved by the Medical Ethics Committee of our hospitals, and patients and their families were informed and signed the informed consent form and completed postoperative follow-up data. Exclusion criteria are as follows: history of preoperative pelvic surgery; severe cardiac, hepatic, and renal insufficiency; preoperative radiotherapy or chemotherapy; preoperative urinary retention; preoperative urinary incontinence of moderate degree or more; and combined mental disorders or psychological disorders.

### 2.1. Surgical Treatment

Both groups underwent extensive laparoscopic hysterectomy+pelvic lymph node dissection under general anaesthesia, performed by the same team of surgeons. After general anaesthesia, the bladder was placed in a cystotomy position, a catheter was left in place, and a cup was placed vaginally; a pneumoperitoneum was established, the pelvic and abdominal cavities were explored, and the trocar was inserted by puncture at the intersection of the lateral umbilicus and the left and right midclavicular lines and at the left and right lateral McKinsey points, respectively, and the pelvic lymph nodes were cleared first, followed by extensive hysterectomy, and the uterus and pelvic lymph nodes were removed vaginally.

### 2.2. Integrated Chinese Medicine Nursing Interventions

In the control group, routine nursing interventions were carried out, such as preoperative and postoperative psychological rehabilitation care to relieve patients' psychological pressure and postoperative strengthening of urinary tract care, keeping the catheter open to prevent urinary tract infection, and timely observation and recording of urine volume, urine colour, and properties; patients were instructed to provide education on functional exercise of the pelvic floor muscles and guidance on functional exercise of the pelvic floor muscles before discharge from the hospital. In the experimental group, technical treatments of traditional Chinese medicine were added to the conventional nursing interventions in the control group. The main interventions were preoperative communication with the patients and postoperative interventions through TCM appropriate techniques (acupuncture+auricular pressure) for a total of two weeks for postradical hysterectomy patients. The patient was treated with acupuncture and auricular pressure on the kidney, Sanyinjiao, subsurface, middle, and Huiyang points, in order to tonify the middle and vital energy, invigorate the meridians, unblock the qi flow of the three jiao organs, and open up the bladder. Ear acupressure is applied to selected acupuncture points such as jiaojiao, Shenmen, bladder, and kidney.

### 2.3. Observation Indicators and Evaluation Criteria

This includes the time of urinary catheter retention, time of first spontaneous urination, time of getting out of bed, and time of anal discharge. Postoperative bladder function recovery and occurrence of urinary retention include bladder function recovery grading, time to bladder recovery, incidence of urinary retention, and residual urine volume after catheter removal. Urogenital tract disorder-related questionnaire (UDI-6) score [19]. Evaluation criteria are as follows: bladder function recovery grading criteria: grade I—residual urinevolume < 50 ml, good bladder function recovery; grade II—residual urine volume of 50-100 ml, slightly poor bladder function recovery; grade III—residual urinevolume > 100 ml, poor bladder function recovery; grade IV—obvious obstruction to urination after removal of urinary catheter in the bladder; grade V—no recovery of bladder function. Good recovery rate = number of patients (bladder function recovery grade I + grade II)/total number of patients.

## 3. Results

### 3.1. Comparison of Postoperative Bladder Function Indicators between the Two Groups of Patients

The time of urinary catheter retention, time of first spontaneous urination, time of getting out of bed, and time of anal venting were all better in the experimental group than in the control group, and the differences were statistically significant (*p* < 0.05); see Table 1.

### 3.2. Comparison of the Incidence of Residual Urine Volume and Urinary Retention between the Two Groups

The rate of good bladder function recovery was higher in the experimental group than in the control group, and the rates of bladder recovery, residual urine volume, and urinary retention were better than those in the control group, with statistically significant differences (*p* < 0.05); see Table 2.

### 3.3. Urinary Index UDI-6 Score and Patient Perception of Urination

After surgery, there was no significant difference in the UDI-6 score between the two groups. 2 weeks after surgery, the UDI-6 score of the experimental group was always lower than that of the control group, and the difference was statistically significant (*p* < 0.05). In addition, after surgery, both groups had difficulty in urination, and there was no significant difference. 2 weeks after surgery, 60 people in the experimental group felt better in urination and 48 people in the control group; the experimental group felt better in urination than the control group; the difference was statistically significant (*p* < 0.05). See Table 3.

## 4. Discussion

In clinical practice, postoperative urinary retention is often prevented and treated by intermittent clamping of urinary catheters, functional exercises for the pelvic floor, bladder irrigation, and potassium permanganate sitz baths [20–22]; Chinese medicine classifies urinary retention under the category of “retention of urine.” The pathogenesis of the disease is mainly due to trauma, which causes damage to the ramifications of the stroke and veins, blockage of the tendons and veins, failure to consolidate the essence and blood, resulting in deficiency of qi and blood, unfavorable qi-transformation of the kidneys and bladder, and failure to open and close the bladder, resulting in blockage of urination [23–25]. The main lesion is in the bladder. It is better to regulate the triple energizer Qi mechanism and dredge the bladder. During radical hysterectomy, when the ureter is free, the nerves in the bladder and lower ureter are partially removed, or the parasympathetic and sympathetic nerves entering and leaving the bladder and urethra are removed together with the main ligament of parauterine tissue and pelvic lymph node, so that the afferent and efferent nerve fibers of the bladder are damaged. The nerve distribution area of S1-S4 sacral nerve can be stimulated through collaterals or meridians, passively inducing the rhythmic systolic and diastolic movement of detrusor and bladder sarcomere and increasing the coordination function between them, reflex stimulation, excitation of spinal cord, and advanced micturition center [26–28]; the external treatment of traditional Chinese medicine is simple and effective. According to the theory of traditional Chinese medicine, the method of pressing needle+auricular point sticking and pressing can be used for treatment and prevention.

The project team consulted the classics and literature and selected Shenshu, Sanyinjiao, CILU, Zhonglu, and Huiyang for the treatment of pressing needle combined with auricular point sticking, so as to achieve the purpose of tonifying middle Qi, dredging meridians and activating collaterals, unblocking triple energizer Qi mechanism, and benefiting bladder. For ear acupoint seed embedding, the project team consulted the classics and literature and selected sympathetic, Shenmen, the bladder, the kidney, and other acupoints for ear acupoint sticking therapy, so as to achieve the functions of promoting Qi, reducing inversion, promoting water and detoxification, autonomously regulating nerve function, tonifying the lower yuan, tonifying the kidney, strengthening yang, moistening, nourishing meridians, and strengthening the body. In the current study, the experimental group was treated with a traditional Chinese medicine characteristic therapy based on routine nursing. We found that the retention time of urinary catheter, the time of first spontaneous urination, the time of getting out of bed, and the time of anal exhaust in the experimental group were better than those in the control group. The recovery rate of bladder function in the experimental group was higher than that in the control group, and the recovery time, residual urine volume, and the incidence of urinary retention in the experimental group were better than those in the control group. The UDI-6 score of the experimental group was better than that of the control group.

In terms of pressing acupuncture points, Shenshu point comes from (LINGSHUBEISHU), which is the acupoint of “foot sun bladder meridian,” which can strengthen the kidney qi and enhance the function of the kidney. Traditional Chinese medicine believes that the kidney governs water and regulates both bowels, which is an important acupoint for regulating water conservancy and Qi [29, 30]. Sanyinjiao is derived from (ZHENJIUJIAYIJING). This point is the intersection point of the three meridians of foot Taiyin spleen meridian, foot Jueyin liver meridian, and foot Shaoyin kidney meridian. Therefore, Sanyinjiao can regulate the liver and spleen and benefit the kidney yin. It has the effects of strengthening the spleen and regulating blood, tonifying the kidney and calming the liver, dredging meridians, and activating collaterals [31]. Ba GUI is derived from the (Yellow Emperor's Canon of internal medicine). Pressing CI Luo points can induce the release of Qi and blood to the anterior yin of the abdomen and bladder, pressing Zhong Luo points can induce the release of forward yin and anus, and pressing CI Luo and Zhong Luo points can dredge the middle Qi, activate blood circulation and remove blood stasis, and have the dual functions of stimulating motor afferent and efferent nerves, so as to achieve the functions of regulating qi and blood, yin, and yang, benefiting official orifices and restoring micturition function [32]. Huiyang point is derived from (ZHENJIUJIAYIJING). It is the intersection of bladder meridian and governor vessel. It has the functions of dredging waist and kidney, warming yang and promoting water, and helping bladder gasification. The afferent nerve of Huiyang point and the afferent nerve innervating bladder overlap multiple ganglion segments. Therefore, it is speculated that pressing Huiyang can regulate bladder function [33]. In addition, as far as the acupoints of embedding seeds in the ear points are concerned, the sympathetic nature is flat, so it has the effects of promoting Qi, reducing stress, and promoting water and detoxification. This point is an important point for visceral analgesia, spasmolysis, and promoting blood circulation to regulate the function of autonomic nerve. Shenmen acupoint belongs to the heart meridian of hand Shaoyin, which can regulate the autonomic nerve, replenish heart qi, stabilize the mind, intersect the heart and kidney, help each other with water and fire, and depend on each other [34]. Bladder point belongs to the bladder meridian of foot sun, which can dredge tendons and relieve surface, clear heat and water, tonify kidney and Qi, dredge collaterals and relieve pain, and is conducive to lower jiao and lower yuan [35]. The kidney ear point belongs to the foot Shaoyin kidney meridian and is useful for tonifying the kidney, strengthening the Yang, penetrating dampness, nourishing the meridians, and strengthening the body [36]. Therefore, comprehensive nursing based on the appropriate technology of traditional Chinese medicine can improve urinary retention and restore bladder function in patients with cervical cancer after hysterectomy.

## Figures and Tables

**Table 1:** Postoperative bladder function indicators in both groups ($\overset{¯}{X}\pm S$).

Group	*n*	Duration of urinary catheter retention (d)	Time to first spontaneous urination (h)	Time out of bed (h)	Anal evacuation time (h)
Experimental group	74	5.45 ± 1.21	4.25 ± 1.32	31.24 ± 4.52	1.25 ± 0.86
Control group	74	6.82 ± 1.43	5.84 ± 1.45	38.62 ± 3.85	1.68 ± 0.75
*t*	/	6.291	6.975	10.692	3.241
*p*	/	0.000	0.000	0.000	0.001

*p* < 0.05 means the difference is statistically significant.

**Table 2:** Incidence of postoperative urinary retention in both groups ($\overset{¯}{X}\pm S/n$, %).

Group	*n*	Bladder function recovery rate	Residual urine volume	Incidence of urinary retention
Experimental group	74	68 (91.89)	75.24 ± 8.65	4 (5.41)
Control group	74	55 (74.32)	91.47 ± 8.72	13 (17.57)
*t*/*x*^2^	/	8.134	11.367	5.383
*p*	/	0.004	0.000	0.020

*p* < 0.05 means the difference is statistically significant.

**Table 3:** UDI-6 scores for voiding indicators in both groups ($\overset{¯}{X}\pm S/n$, %).

	*n*	UDI-6 scores		Excellent rate of urinary sensation
		Postoperative	Two weeks after surgery	Two weeks after surgery
Experimental group	74	35.45 ± 4.21	25.65 ± 2.51	60 (81.08)
Control group	74	36.41 ± 4.15	32.47 ± 3.85	48 (64.86)
*t*/*x*^2^	/	1.396	12.765	4.933
*p*	/	0.164	0.000	0.026

*p* < 0.05 means the difference is statistically significant.

## Data Availability

The datasets used and analyzed during the current study are available from the corresponding author upon reasonable request.

## References

[1] Olusola P., Banerjee H. N., Philley J. V., Dasgupta S. (2019). Human papilloma virus-associated cervical cancer and health disparities. *Cell*.

[2] Cancer Genome Atlas Research Network (2017). Integrated genomic and molecular characterization of cervical cancer. *Nature*.

[3] Marnitz S., Tsunoda A. T., Martus P. (2020). Surgical versus clinical staging prior to primary chemoradiation in patients with cervical cancer FIGO stages IIB-IVA: oncologic results of a prospective randomized international multicenter (Uterus-11) intergroup study. *International Journal of Gynecological Cancer*.

[4] Poddar P., Maheshwari A. (2021). Surgery for cervical cancer: consensus & controversies. *The Indian Journal of Medical Research*.

[5] Bujnak A. C., Tewari K. S. (2021). Should adjuvant chemotherapy be formally studied among patients found to have pelvic lymph node metastases following radical hysterectomy with lymphadenectomy for early-stage cervical cancer?. *Journal of Gynecologic Oncology*.

[6] Leetanaporn K., Hanprasertpong J. (2019). Impact of obesity on clinical outcomes in patients with early-stage cervical cancer after radical hysterectomy with pelvic node dissection. *Oncology Research and Treatment*.

[7] Li H., Zhou C.-K., Song J. (2019). Curative efficacy of low frequency electrical stimulation in preventing urinary retention after cervical cancer operation. *World Journal of Surgical Oncology*.

[8] Mengatto M. F., Castro B. G. R., Nobrega L. (2020). Early removal of indwelling urinary catheter after radical surgery for early-stage cervical cancer—a cohort study. *Journal of Surgical Oncology*.

[9] Kowalik U., Plante M. K. (2016). Urinary retention in surgical patients. *Surgical Clinics of North America*.

[10] Derks M., van der Velden J., Frijstein M. M. (2016). Long-term pelvic floor function and quality of life after radical surgery for cervical cancer: a multicenter comparison between different techniques for radical hysterectomy with pelvic lymphadenectomy. *International Journal of Gynecological Cancer*.

[11] Gelber J., Singh A. (2021). Management of acute urinary retention in the emergency department. *Emergency Medicine Practice*.

[12] Ghuman A., Kasteel N., Karimuddin A. A., Brown C. J., Raval M. J., Phang P. T. (2018). Urinary retention in early urinary catheter removal after colorectal surgery. *American Journal of Surgery*.

[13] Zheng C., Li Z., Lu H., Zhou Y. (2021). Effectiveness of acupuncture on urinary retention: a meta-analysis. *Evidence-Based Complementary and Alternative Medicine*.

[14] Zhong Y., Zeng F., Li J., Yang Y., Zhong S., Song Y. (2018). Electroacupuncture for postoperative urinary retention: a systematic review and meta-analysis. *Evidence-Based Complementary and Alternative Medicine*.

[15] Chen S., Sun H., Xu H., Zhang Y., Wang H. (2020). Effects of acupuncture on hospitalized patients with urinary retention. *Evidence-Based Complementary and Alternative Medicine*.

[16] Lauterbach R., Ferrer Sokolovski C., Rozenberg J., Weissman A. (2018). Acupuncture for the treatment of post-partum urinary retention. *European Journal of Obstetrics, Gynecology, and Reproductive Biology*.

[17] Zhao Q., Yan C., Dan M., Jia H. (2021). Efficacy and safety of acupuncture for urinary retention after hysterectomy: a systematic review and meta-analysis. *Medicine*.

[18] Ruengwongroj P., Muengtaweepongsa S., Patumanond J., Phinyo P. (2020). Effectiveness of press needle treatment and electroacupuncture in patients with postherpetic neuralgia: a matched propensity score analysis. *Complementary Therapies in Clinical Practice*.

[19] Mikuš M., Ćorić M., Matak L., Škegro B., Vujić G., Banović V. (2020). Validation of the UDI-6 and the ICIQ-UI SF–Croatian version. *International Urogynecology Journal*.

[20] Zong J., You M., Li C. (2022). Effect of Kegel pelvic floor muscle exercise combined with clean intermittent self-catheterization on urinary retention after radical hysterectomy for cervical cancer. *Pakistan Journal of Medical Sciences*.

[21] Jaffar A., Mohd Sidik S., Foo C. N., Muhammad N. A., Abdul Manaf R., Suhaili N. (2022). Preliminary effectiveness of mHealth app-based pelvic floor muscle training among pregnant women to improve their exercise adherence: a pilot randomised control trial. *International Journal of Environmental Research and Public Health*.

[22] Santa Mina D., Au D., Alibhai S. M. H. (2015). A pilot randomized trial of conventional versus advanced pelvic floor exercises to treat urinary incontinence after radical prostatectomy: a study protocol. *BMC Urology*.

[23] Wu D., Tang H. X., Wu Y., Qian S. B., Xu D., Qi J. (2020). The possible association between serum interleukin 8 and acute urinary retention in Chinese patients with benign prostatic hyperplasia. *Andrologia*.

[24] Wang S., Wang M., Zhang H. (2021). Effect observation on modified Zishen Tongguan decoction combined with acupuncture in treatment of urinary retention after cervical cancer surgery and its influence on the incidence of adverse reactions. *Evidence-Based Complementary and Alternative Medicine*.

[25] Lin S.-K., Lin P.-H., Hsu R.-J., Chuang H.-C., Liu J.-M. (2017). Traditional Chinese medicine therapy reduces the catheter indwelling risk in dementia patients with difficult voiding symptoms. *Journal of Ethnopharmacology*.

[26] Karani R., Mahdy A., Asghar F. (2020). Postoperative urinary retention in patients who undergo joint arthroplasty or spine surgery. *JBJS Reviews*.

[27] do Nascimento Ceratti R., Beghetto M. G. (2021). Incidence of urinary retention and relations between patient’s complaint, physical examination, and bladder ultrasound. *Revista Gaúcha de Enfermagem*.

[28] Szymański J. K., Słabuszewska-Jóźwiak A., Jakiel G. (2021). Fowler’s syndrome-the cause of urinary retention in young women, often forgotten, but significant and challenging to treat. *International Journal of Environmental Research and Public Health*.

[29] Wang S.-C., Jiang Y.-M., Qiu L.-R., Su M. (2021). Efficacy of needling acupoints of Guanyuan (CV4), Sanyinjiao (SP6), Zusanli (ST36), Pishu (BL20), Shenshu (BL23), Zigong (EX-CA1) on expression of p38 mitogen-activated protein kinase in ovarian tissue in rats with premature ovarian failure induced by cyclophosphamide. *Journal of Traditional Chinese Medicine*.

[30] Takeda A., Koike T., Urata S., Ishida T., Oshida Y. (2018). Effect of acupuncture at acupoint of Shenshu (BL 23) on the bones of ovariectomized rats. *Journal of Traditional Chinese Medicine*.

[31] Wang Z.-J., Zhang Y., Guo W. (2020). Is single acupoint Sanyinjiao (SP 6) effective in managing insomnia? A systematic review of randomized controlled trials. *Global Health Medicine*.

[32] Kim J.-H., Han J.-Y., Park G.-C., Lee J.-S. (2019). Effects of electroacupuncture combined with computer-based cognitive rehabilitation on mild cognitive impairment: study protocol for a pilot randomized controlled trial. *Trials*.

[33] Liu Y., Liu L., Wang X. (2013). Electroacupuncture at points Baliao and Huiyang (BL35) for post-stroke detrusor overactivity. *Neural Regeneration Research*.

[34] Wu P., Cheng C., Song X. (2020). Acupoint combination effect of Shenmen (HT 7) and Sanyinjiao (SP 6) in treating insomnia: study protocol for a randomized controlled trial. *Trials*.

[35] Shen J., Luo R., Zhang L., Li Y., Ke L., Gao Z. (2019). Using electroacupuncture with optimized acupoint positioning to predict the efficacy of sacral neuromodulation of refractory overactive bladder: a case report. *Medicine (Baltimore)*.

[36] Mao J. J., Liou K. T., Baser R. E. (2021). Effectiveness of electroacupuncture or auricular acupuncture vs usual care for chronic musculoskeletal pain among cancer survivors. *Oncologia*.

